# Investigation and Discrimination of Ballpoint Pen Inks by Analytical Techniques and Chemometrics

**DOI:** 10.1155/2022/7450539

**Published:** 2022-08-12

**Authors:** Mehwish Sharif, Sohail Chand, Syed Azhar Ali Shah Tirmazi, Umar Farooq, Muhammad Makshoof Athar, Madeeha Batool

**Affiliations:** ^1^School of Chemistry, University of the Punjab, Lahore 54590, Pakistan; ^2^College of Statistical and Actuarial Sciences, University of the Punjab, Lahore 54590, Pakistan

## Abstract

A population study has been performed for Pakistani ballpoint pen inks of blue, black, red, and green colors (a total of four colors) commercially used in Pakistan. Ballpoint pen inks have been investigated and discriminated by using UV/Vis spectroscopy and FTIR spectroscopy. We have calculated and compared the results in terms of discriminating power (DP). The statistical techniques of principal component analysis and cluster analysis have been applied on obtained data. By visual comparison, the best DP is obtained for green ballpoint pen inks, i.e., 0.866 by using UV/Vis spectroscopy and FTIR techniques. Black and red ballpoint pen inks showed the highest DPs by using UV/Vis spectroscopy; however, blue ballpoint pen inks got the highest DP by using FTIR spectroscopy. DP has been improved by using chemometric techniques and higher DPs are obtained as compared to visual examination.

## 1. Introduction

Writing instruments are continuously used to mark and sign official documents to authenticate them even in the recent era of technology wherever printers, scanners, and other digital devices have abridged the use of documents written with hand [1]. The probability of deceit in handwritten documents is greater in developing countries [2]. In most of the questioned document cases involving ink, the ballpoint pen ink used is the main evidence for determining that document is genuine or forged. Ballpoint inks have a very complex chemical composition that is necessary for its better quality and color. Ballpoint pen inks consist of solvents, pigments, dyes, lubricants, emulsifiers, pH buffers, biocides, and resins [3, 4]. Among these components, dyes and pigments or their combinations have an important role in the identification/comparison of inks as they remain on paper for a very long duration [5].

Before 1950, the analytical techniques used for ink analysis were very simple requiring specific sample preparation and therefore were time consuming [6]. Before the 1970s, the interpretations of methods were relying on only expert knowledge. In 1970, the modern scientific methods have been used for the analysis of questioned documents. After the 1990s, the spectroscopic methods were started for nondestructive and destructive analysis of suspected documents [7, 8]. For destructive methods, the paper surface with ink is punched and examined, whereas no specific preparation of the sample is required for the nondestructive examination of ink and hence integrity of the document is conserved [9, 10].

The destructive methods used for determination of makeup of ballpoint inks chemically include Fourier transform infrared spectroscopy (FTIR) [9, 11, 12], thin layer chromatography (TLC) [11, 13], UV/Vis spectroscopy [5, 11, 12, 14], mass spectroscopy [14, 15], and high performance liquid chromatography (HPLC) [16–18]. Nondestructive methods used by document examiners are luminescence spectroscopy [10], infrared spectroscopy [4, 19, 20], and Raman spectroscopy [4, 9, 19, 21, 22]. These techniques can differentiate and characterize samples of a ballpoint in a small number without damaging. Raman spectroscopy and FTIR give knowledge about the chemical composition for ballpoint ink, e.g., dyes, resins, and solvents, and therefore assists in the characterization of forensic samples of ink.

These methods are time consuming when used for a large number of samples, and for that reason they need the inclusion of statistical methods combined with analytical methods. Consequently, from the last few decades in forensic science, a mixture of analytical methods along with the statistical applications have been continuously used.

In our research, the analysis of ballpoint pen inks is performed destructively. The results are reported in terms of discriminating power (DP). The DP of an item describes how rapidly the change occurs from low probability to high probability of the right response. A highly discriminating item gives better results having a very less chance of ambiguity. Using DP, a comparison of two items can be made directly to determine which can better calculate a particular attribute [23]. It is calculated according to the following formula [24]:

(1) $$\begin{array}{c} \text{DP}=\frac{\text{number of discriminating sample pair}}{\text{number of possible sample pair}}. \end{array}$$

The obtained data are evaluated using statistical techniques, i.e., principal component analysis (PCA) and cluster analysis. PCA is a dimension-reduction statistical technique that is used to decrease a large set of variables to a small set that still has nearly all of the information in the large set. Two subsequent approaches for discrimination of ballpoint ink samples, i.e., destructive UV/Vis spectroscopy and FTIR spectroscopy, have been represented in terms of cumulative variance (%). Cluster analysis is the classification of data objects into similar groups based on their defined distance measurements. Cluster analysis is used in different fields, e.g., data mining, machine learning, pattern recognition, systems biology, genomics, image analysis, etc. Cluster analysis is performed by R. R is a programming language and software environment for statistical computing and graphics supported by the R Foundation for statistical computing. The R language is frequently applied amongst statisticians and data miners for data analysis and development of statistical software.

The purpose of the present work is to differentiate between different ballpoint pen inks commercially used in Pakistan to examine alteration and counterfeiting in documents in forensic science using UV/Vis spectroscopy and FTIR spectroscopy techniques with the help of chemometrics. The present research study will be very valuable for forensic document examiners in convincing the law enforcement community that ink is evidence of scientific importance. Moreover, this study will be helpful for the creation of an ink database of different ballpoint pen inks based on UV/Vis spectroscopy and FTIR spectroscopy, as there is no database for the Pakistani ballpoint pen inks. Hence, the examination of Pakistani ballpoint pen inks and application of chemometrics (PCA and cluster analysis using R) on spectral data is new.

## 2. Experimental

### 2.1. Chemical Reagents

Ethanol and methanol of HPLC grade are purchased from Sigma-Aldrich, Singapore.

### 2.2. Samples Preparation

A total of 55 ballpoint pen ink samples as mentioned in Table 1 (20 different brand names of blue ballpoint pen inks, 19 different brand names of black ballpoint pens inks, 8 different brand names of red ballpoint pens inks, and 6 different brand names of green ballpoint pens inks) commercially used in Pakistan were obtained from different stationery stores in Lahore, Pakistan in 2017. Each of the ballpoint pen ink has been primarily applied on a separate A4 paper, white color with weight 80 g/m^2^. The sample was allowed to dry for 12 hours. The samples were dried to keep away from the transfer of a sample of ink from one paper to adjacent papers. In this way, false-positive results are avoided. The same procedure was used for all samples using the same size of paper. The samples were kept in normal environmental conditions at 25°C to 27°C without direct exposure to light in a dark wooden box. Each ballpoint pen ink sample was punched with the help of Deluxe Aluminum Harris Micro-Punch (1 mm), Electron Microscopy Sciences, Hatfield, PA, USA. The extraction of ink from the paper was performed using ethanol: methanol in mixture (70 : 30) as a solvent in glass vials. For reproducibility, six different extractions or samples were made using different writing micro plugs of the same ink in separate vials. Blank A4 size paper was also mixed with ethanol: methanol mixture as a solvent to calculate the effect of matrix on sampling.

### 2.3. UV/Visible Spectroscopy

Preparation of samples intended for UV/Vis spectroscopy was done using punching 25 micro plugs of paper bearing writing with the help of Harris Aluminum Micro-Punch of the size of 1 mm. Each of these micro plugs was dissolved in 120 *μ*L ethanol: methanol mixture in a separate sample vial. For UV/Vis analysis, T90 + UV/VIS spectrophotometer, PG Instruments Limited, Beijing, China, was utilized. The spectral range for recording results was full scan, i.e., 190–800 nm with scan speed of 1000 nm/min. Quartz cell of path length 1 cm was used. For data processing, UVWin 5 spectrophotometer software was used.

### 2.4. FTIR Spectroscopy

The spectra were acquired using Carry 630 FTIR spectrometer, Agilent Technologies, USA, equipped with a diamond ATR sampling interface. Samples were analyzed by collecting 32 scans at 2 cm^−1^ spectral resolution over a spectral range of 4,000 cm^−1^–650 cm^−1^. Agilent Micro Lab PC software, automated IQ/OQ, 21CFR Part 11 compliant, resolutions Pro for advanced data analysis was used for FTIR analysis.

Ten microliter of extracted ballpoint inks has been applied directly onto the diamond ATR accessory. For better results, the prepared ink sample was directly applied on a crystal of diamond, independent of the amount but enough to cover the area of crystal [25].

### 2.5. Softwares Used

1. Origin software (Version 6.0) is used to draw and normalize graphs in this research study for visual analysis.
2. SPSS version 23 is used for PCA.
3. R Core Team (2020). R is a language and environment for statistical computing, R Foundation for statistical computing, Vienna, Austria. R is used for cluster analysis.

## 3. Results and Discussion

### 3.1. UV/Vis Spectroscopy

For ink's coloring agents, UV/Vis spectroscopy is a principle investigation tool [26]. Ballpoint inks discrimination is considered based on qualitative analysis of absorption spectra. Minor differences in peak positions and relative intensities contribute to ballpoint inks differentiation.

Sample pairs are defined as blue ballpoint ink sample B1 paired with blue ballpoint ink sample B2, then B1 with B3, B1 with B4, and similarly B1 with B5, B6, B7, B8, B9, B10, B11, B12, B13, B14, B15, B16, B17, B18, B19, and B20. Then pairing of B2 is started with B3, B4, B5, B6, B7, B8, B9, B10, B11, B12, B13, B14, B15, B16, B17, B18, B19, and B20. Then pairing of B3 is started with B4, B5, B6, B7, B8, B9, B10, B11, B12, B13, B14, B15, B16, B17, B18, B19, and B20. In this way, all blue ballpoint ink samples are paired. Black, red, and green ballpoint ink samples are paired in a similar way.

Sample pairs showing peaks at the same position for UV/Vis spectrum and FTIR spectrum are nondiscriminating sample pairs and sample pairs showing peaks at different positions UV/Vis spectrum and FTIR spectrum are discriminating sample pairs.

For proper representation of 20 inks of blue ballpoint pens used in this study, the samples are divided into three groups based on obtained UV/Visible spectra (Figure 1). Samples are divided into groups on the basis of obtained UV/Vis spectra. Samples with peaks at the same position are grouped into one group and samples with different peaks at different positions are grouped into different groups. Group I consists of B1, B2, B3, B5, B6, B7, B9, B11, B14, B15, and B18; group II comprised of only B8; and group III consists of B4, B10, B12, B13, B16, B17, B19, and B20.

The total number of possible pairs calculated visually for blue ballpoint pen inks is 190, out of which 107 are discriminating pairs and the remaining 83 are nondiscriminating pairs. Calculated DP for blue ballpoint inks using UV/Vis technique is 0.563.

In a similar way, 19 black ballpoint inks are divided into five groups (Figure 2). Group I comprised of K2, K4, and K15; group II included K1, K11, and K13; group III consisted of K3, K5, K6, K10, and K14; group IV comprised of K8, K9, K12, K16, K17, and K19; and group V is composed of K7 and K18. Similarly, for 19 black ballpoint inks, the total number of possible pairs is 171, out of which 139 are discriminating pairs and number of nondiscriminating pairs is 32. DP calculated using the UV/Vis technique for black ballpoint inks is 0.812.

For red ballpoint inks, three groups are suggested (Figure 3). Group I includes R1, R4, and R6; group II includes R2, R3, R5, and R8; and group III includes only R7. For red ballpoint inks, the calculated total number of possible pairs is 28, including 19 discriminating and 9 nondiscriminating sample pairs, resulting in DP of 0.678.

Four groups have been devised for green ballpoint inks used in this study (Figure 4). Group I consists of only sample G2, group II consists of samples G1 and G3, group III consists of G5, and group IV consists of samples G4 and G6. For green ballpoint inks used in this study, the total number of calculated possible sample pairs is 15, consisting of 13 discriminating sample pairs and 2 nondiscriminating sample pairs. The calculated DP is 0.866 for green ballpoint inks using UV/Vis spectroscopy.

Ballpoint ink samples have been analyzed six times for the evaluation of repeatability of the obtained results. Comparable results have been acquired as compared with ballpoint inks samples extracted from the surface of the paper in a solvent. The relative standard deviation (RSD) observed in this study was 3%. Knowledge of DP is necessary for interpretation of results as only partial information is available in the literature [27, 28]. For this study, the calculated DP is 0.563 for blue ballpoint inks which is lower as compared to the literature DP value 0.71 [29] for blue pen inks.

### 3.2. FTIR Spectroscopy

FTIR is a technique used to discriminate ballpoint pen inks based on the presence of different solvents, dyes, or resins. FTIR spectrum in the range of 400–2000 cm^−1^ provides sufficient information about chemical ingredients of samples of the ink, e.g., dyes, resins, and solvents. In this study, most of the ballpoint ink samples (blue, black, red, and green) showed peaks at around 1500–1700 cm^−1^, 1000–1400 cm^−1^, 910 cm^−1^, and 700 cm^−1^.

The differentiation of inks of ballpoint pens by using FTIR spectra has been completed because of the differentiation for the number of peaks, their position, and their intensities [30]. There are two regions of an IR spectrum: i.e., functional group region (above 1500 cm^−1^) helps in the identification of different functional groups and fingerprint region (below 1500 cm^−1^) helps in the characterization of the whole molecule.

In the current research, the discrimination of ballpoint pen inks by FTIR spectra was attained based on a qualitative comparison of spectra for analyzed samples. In the sampling of ballpoint pen inks, the age of ballpoint pen inks was not managed, and the ratios of intensity were not considered for the differentiation of ballpoint pen inks [9, 31].

The region between 1800 and 650 cm^−1^ is considered as the most important region for ballpoint pen ink analysis [32] and most variability exists in the 650–1800 cm^−1^. Transmittance peak positions are compared with reference peak positions in the literature; e.g., the peaks at 1585 cm^−1^ and 1170 cm^−1^ are characteristics of ballpoint pen inks [33] and are attributed to the triarylmethane dyes [34]. By using a qualitative approach in FTIR spectra for blue ballpoint inks, four groups are obtained (as shown in Figure 5). B1, B2, B5, B6, B10, B11, B12, B14, B17, B18, B19, and B20 are placed in group I; B4, B15, and B16 in group II; B3, B7, B8, and B9 in group III; and B13 in group IV. By using a qualitative approach in FTIR spectra for blue ballpoint inks, DP calculated visually for inks of blue ballpoint pens is 0.605 based on 190 total number of sample pairs, 115 discriminating sample pairs, and 75 nondiscriminating sample pairs (Table 2). The RSD observed in this study was 3%.

Four groups are devised for black ballpoint inks used for this study as mentioned in Figure 6. Group I includes K1, K2, K3, K4, K6, K8, K9, K10, K13, K14, K15, K17, K18, and K19; group II includes K5, K7, and K12; group III includes only K11; and group IV includes K16. For black ballpoint inks, the total number of possible sample pairs is 171; discriminating pairs are 76 and nondiscriminating pairs are 95, resulting in DP of 0.444 as mentioned in Table 2.

Red ballpoint inks in this study are divided into four groups as mentioned in Figure 7. Group I includes R1, R2, R3, R4, and R6; group II consists of R5; group III consists of R7; and group IV includes R8. Red ballpoint inks in this study show the total number of possible sample pairs is 28 (18 discriminating and 10 nondiscriminating) resulting in DP of 0.642. For green ballpoint inks using FTIR, four groups are devised (Figure 8). G1 and G3 are included in group I; G2 in group II; G5 in group III, and G4 and G6 in group IV. For green ballpoint inks using FTIR, the total number of possible samples is 15 ; 13 discriminating and 2 nondiscriminating. The calculated DP by using FTIR with green ballpoint pen inks is 0.866 as mentioned in Table 2.

Based on the qualitative information, DP for this research study by using FTIR spectroscopy has been found as 0.605 for blue, 0.444 for black, 0.642 for red, and 0.866 for green colored inks.

The DP for ballpoint pen ink is 0.563, 0.812, 0.678, and 0.866 for blue, black, red, and green inks, respectively, by UV/Vis spectroscopy and DP is 0.605, 0.444, 0.642, and 0.866 for blue, black, red and green ballpoint pen inks, respectively, by using FTIR spectroscopy. Green ballpoint pen inks show the highest DP, i.e., 0.866 and DP is the same by using UV/Vis spectroscopy and FTIR spectroscopy. Therefore, green ballpoint pen inks should be used for high profile matters in which chances of forgery/fraud are maximum. Table 2 comes with DP values obtained from visual comparison of spectra drawn from UV/Vis spectroscopy and FTIR spectroscopy data.

### 3.3. Statistical Analysis

For the statistical representation of large spectral data for ballpoint pen inks in this study, we have used factor analysis with principal components as an extraction method. We have also used Varimax rotation with Kaiser Normalization for the selection of the important principal components for further analysis.

Row scaling method was used for normalization [3]. The normalization resolves the problem of variations in the amount of the samples used to prepare the ink writing and after normalization, the spectra can be compared. Moreover, the rotation of principal components allows us to have a simplified structure for better understanding and interpretation.

PCA [35] uses linear combinations of the original variables (patent variables) to define new variables called principal components or PCs (latent/hidden variables) which leads to dimension reduction. Thus, it decreases the number of variables required for the measurement of objects in a dataset and also identified principal components that help to study the structure of variables grouped based on their correlations. Ideally, the extraction of principal components is such that the first principal component explains the largest variation in the original data. A certain proportion of the remaining unexplained variance is explained by the extraction of the second principal component. The process of extraction can be repeated *m* times for *m* patent variables until all the variation of the original variables is explained by the principal components. According to the definition, the components extracted are orthogonal and consequently show no correlation with each other. Only with the extraction of the first two or three principal components, one can project the objects of a dataset on a plane or in a three-dimensional space, respectively, and imagine an otherwise insignificant *m*-dimensional space [14].

The associations of the principal component scores with the original scores on the m patent variables are called component loadings and are the basis for the qualitative interpretation of the components extracted. The Varimax rotation technique is used to make sure that the loading of a patent variable is maximized on one component while it is minimized on all other components. The process makes the interpretation easier for the principal components. Original variables are expected to load highly on the same component if original variables have already been correlated. Characterization of each extracted component has been made by its eigenvalue which almost relates to the number of patent variables this component shows. Two criteria have been used for a number of principal components extracted from a given dataset: the Kaiser criterion and the scree plot. Following the Kaiser criterion [25], only components with eigenvalues greater than 1 are supposed to be extracted; the underlying principal is that components showing less than one variable should not be considered. Conversely, a scree plot is used to show the proportion of the total variation in a dataset that is clarified by each of the components in PCA. With the help of a scree plot, we can determine the number of components required to summarize the data. In the scree plot, the principal component number is shown on the *x*-axis and corresponding eigenvalues on the *y*-axis. The position where the slope of the curvature is noticeably leveling off (the ‘elbow) specifies the number of factors that should be produced by the analysis. Away from this point, no additional progress in explanation of variance could be made and additional components are not required.

After factor analysis, it has been found that a 100% variation of the data is explained by all the principle components. But according to Kaiser Criteria, from all the principal components, the first two principal components explain almost all variation in the original variables. For FTIR spectroscopy, the cumulative variance (%) is highly significant that is 94.227, 95.787, 98.893, and 96.935 for blue, black, red, and green ballpoint pen inks, respectively, as mentioned in Table 3. In a similar way, the cumulative variance (%) for UV/Vis spectroscopy is also very significant, i.e., 98.872, 98.519, 99.092, and 98.197 for blue, black, red, and green ballpoint pen inks, respectively (Table 3).

The Varimax rotation maximizes the natural loading and minimizes the offloading, without changing the relations between the data (independent component). Therefore, after rotation, the percent of variance per PCs is altered concerning the initial solution. On the other hand, the total variance explained remains equal for the initial solution.

Cluster analysis is performed for UV/Vis spectroscopy and FTIR spectroscopy data using R. Similar types of spectral signatures were observed for some samples of inks by visual inspection which could only be differentiated by multivariate analysis. From cluster analysis of UV/Vis spectroscopy data of blue ballpoint inks, the ballpoint pen ink samples have been divided into two clusters. Cluster 1 consists of ballpoint ink samples 1, 3, 4, 5, 6, 9, 14, and 18. Cluster 2 consists of samples 2, 7, 8, 10, 11, 12, 13, 15, 16, 17, 19, and 20 (as shown in Figure 9). Similarly, cluster analysis of UV/Vis spectroscopy data for black ballpoint inks results in two clusters (Figure 10). Ballpoint ink samples 1, 2, 4, 5, 6, 7, 11, and 13 are in cluster 1 while samples 3, 8, 9, 10, 12, 14, 15, 16, 17, 18, and 19 are in cluster 2.

Two clusters have also been obtained for UV/Vis spectroscopy data of green ballpoint inks. The ballpoint ink samples 1, 3, 4, and 6 come in cluster 1 and samples 2, and 5 come in cluster 2 (Figure 11). In a similar way, UV/Vis spectroscopy data of red ballpoint inks also result in two clusters (as shown in Figure 12). Cluster 1 consists of ballpoint ink samples 1, 3, 4, 7, and 8 and cluster 2 consists of samples 2, 5, and 6.

For cluster analysis of FTIR spectroscopy data of blue ballpoint inks, the two clusters have been obtained. Ballpoint ink samples 1, 2, 3, 7, 8, 9, 14, and 19 come in cluster 1 and samples 4, 5, 18, 6, 10, 11, 12, 13, 15, 16, 17, and 20 in cluster 2 (as shown in Figure 13). Similarly, by cluster analysis of FTIR spectroscopy data for black ballpoint inks, the two clusters have been obtained (as shown in Figure 14). Ballpoint ink samples 1, 2, 6, 11, 12, 13, 14, 16, 17, and 19 are divided in cluster 1 and samples 3, 4, 5, 7, 8, 9, 10, 15, and 18 are divided in cluster 2.

For FTIR spectroscopy data of green ballpoint inks, the two clusters have also been obtained. Ballpoint ink samples 1, 2, 3, and 5 come in cluster 1 and samples 4 and 6 in cluster 2 (Figure 15). For FTIR spectroscopy data of red ballpoint inks, the two clusters have been obtained (as shown in Figure 16). Ballpoint ink samples 1, 2, and 7 come in cluster 1 while samples 3, 4, 5, 6, and 8 in cluster 2.

DP for sample pairs within a cluster has been calculated with the understanding of discriminating and nondiscriminating sample pairs. The sample pairs which have different Euclidean distance have been considered as discriminating sample pairs and sample pairs which are superimposable showing zero Euclidean distance have been considered as nondiscriminating sample pairs.

Some sample pairs of UV/Vis spectroscopy data for blue ballpoint pen inks have not been discriminated against due to the presence of similar types of ink constituents. Therefore, in cluster 2 of blue ballpoint pen inks, out of 66 sample pairs of ink, only two pairs, i.e., 12, 13 and 19, 20, were not discriminated. These sample pairs are superimposable to each other which indicates that they are chemically similar.

Likewise, cluster 2 of black ballpoint pen inks contains 55 ink samples. Among them only one sample pair, i.e., 12, 14, was not differentiated as shown in Table 4.

It is inferred from the above-mentioned discussion that cluster 2 for blue and black ballpoint pen inks shows 0.96 and 0.98 DP, respectively. Therefore, on the whole, discrimination obtained by UV/Vis spectroscopy (destructive approach) for blue ballpoint pen inks is 98% (both cluster's average as mentioned in Table5) and for the black ballpoint pen inks is 99% (average of both clusters) which demonstrates that better results have been obtained as compared to visual comparison of spectra. Similarly, discrimination obtained by UV/Vis spectroscopy (destructive approach) is 100% (both cluster's average, Table 5) for green and red ballpoint pen inks which also shows highly significant results as compared to visual comparison of spectra in which these variations were unnoticed.

From FTIR data cluster analysis data, it is observed that blue ballpoint pen inks contain 66 sample pairs. Out of 66, only one sample pair, i.e., 5, 18, was not differentiated as shown in Table 6. DP for FTIR data of blue ballpoint pen inks is 99% (average of both clusters, Table 5). Discrimination achieved by FTIR spectroscopy (by destructive method) is 100% (both cluster's average) for black, green, and red ballpoint pen inks as shown in Table 5 which also demonstrates better results as compared to visual comparison of spectra. According to research reported by Causin [11], application of chemometrics on FTIR spectroscopy data gives better DP as compared to UV/Vis spectroscopy data. FTIR spectra appear due to presence of resins and solvents in addition to color imparting components.

A table of comparison of ballpoint pen inks for already reported studies and the present study has been made (Table 7). In the table, samples analyzed by using various techniques with or without the help of statistical techniques are summarized. The discrimination calculated in the current study is better as compared to already reported literature studies.

## 4. Conclusions

It is concluded that 55 samples of ballpoint pen ink (20 blue, 19 black, 8 red, and 6 green colors) were differentiated based on UV/Vis spectroscopy and FTIR spectroscopy by using chemometrics.

The DP data for dissimilar analytical techniques or the succession of techniques utilized for Pakistani inks of ballpoint is not obtainable in the literature. In this study, the calculated DP by visual comparison for ballpoint pen ink was 0.563, 0.812, 0.678, and 0.866 for blue, black, red, and green ballpoint inks, respectively, utilizing UV/Vis spectroscopy. Calculated DP for ballpoint pen inks was 0.605, 0.444, 0.642, and 0.866 for blue, black, red, and green inks, respectively, by the use of FTIR spectroscopy.

In short, green color ballpoint pen inks available in Pakistan give better discrimination results compared to blue, black, and red color ballpoint pen inks. Green color ballpoint pen inks give the same DP with UV/Vis spectroscopy and FTIR spectroscopy. However, blue color ballpoint gives good discriminating results using FTIR spectroscopy while black and red color ballpoint pen inks give good discriminating results using UV/Vis spectroscopy, only. Therefore, it is suggested to use green ballpoints for official documentation in Pakistan, to minimize fraudulence. By using chemometric techniques of PCA and cluster analysis, DP has been improved and more significant results are obtained.

The calculated DP is 0.98, 0.99, 1.0, and 1.0 by using the chemometric technique on UV/Vis spectroscopy data for blue, black, red, and green ballpoint inks, respectively. These results are highly significant as compared to examination of the UV/Vis spectra visually, i.e., 0.563, 0.812, 0.678, and 0.866 for blue, black, red, and green ballpoint inks, respectively. Calculated DP was 0.99, 1.0, 1.0, and 1.0 for blue, black, red, and green inks, respectively, by the use of the chemometric technique on FTIR spectroscopy data. These results are also better as compared to visual examination of the FTIR spectra, i.e., 0.605, 0.444, 0.642, and 0.866 for blue, black, red, and green ballpoint inks, respectively.

Further recommended study is the estimation of metal content in blue, black, red, and green ballpoint pen inks, for their discrimination in a better way.

## Figures and Tables

**Figure 1:** UV/Vis spectra for groups I, II, and III of blue ballpoint pen inks.

**Figure 2:** UV/Vis spectra for groups I, II, III, IV, and V of black ballpoint pen inks.

**Figure 3:** UV/Vis spectra for groups I, II, and III of red ballpoint pen inks.

**Figure 4:** UV/Vis spectra for groups I, II, III, and IV of green ballpoint pen inks.

**Figure 5:** FTIR spectra for groups of I II, III, and IV blue ballpoint pen inks.

**Figure 6:** FTIR spectra for groups I, II, III, and IV of black ballpoint pen inks.

**Figure 7:** FTIR spectra for groups I, II, III, and IV of red ballpoint pen inks.

**Figure 8:** FTIR spectra for groups I, II, III, and IV of green ballpoint pen inks.

**Figure 9:** Cluster analysis for UV/Vis spectroscopy data for blue ballpoint pen inks.

**Figure 10:** Cluster analysis for UV/Vis spectroscopy data for black ballpoint pen inks.

**Figure 11:** Cluster analysis for UV/Vis spectroscopy data for red ballpoint pen inks.

**Figure 12:** Cluster analysis for UV/Vis spectroscopy data for green ballpoint pen inks.

**Figure 13:** Cluster analysis for FTIR spectroscopy data for blue ballpoint pen inks.

**Figure 14:** Cluster analysis for FTIR spectroscopy data for black ballpoint pen inks.

**Figure 15:** Cluster analysis for FTIR spectroscopy data for red ballpoint pen inks.

**Figure 16:** Cluster analysis for FTIR spectroscopy data for green ballpoint pen inks.

**Table 1:** Samples of ballpoint pen inks of different colors and brands with sample codes.

Sr. No.	Blue		Black		Red		Green	
	Ink sample	Sample code	Ink sample	Sample code	Ink sample	Sample code	Ink sample	Sample code
1	Sample 1	B1	Sample 1	K1	Sample 1	R1	Sample 1	G1
2	Sample 2	B2	Sample 2	K2	Sample 2	R2	Sample 2	G2
3	Sample 3	B3	Sample 3	K3	Sample 3	R3	Sample 3	G3
4	Sample 4	B4	Sample 4	K4	Sample 4	R4	Sample 4	G4
5	Sample 5	B5	Sample 5	K5	Sample 5	R5	Sample 5	G5
6	Sample 6	B6	Sample 6	K6	Sample 6	R6	Sample 6	G6
7	Sample 7	B7	Sample 7	K7	Sample 7	R7	—	—
8	Sample 8	B8	Sample 8	K8	Sample 8	R8	—	—
9	Sample 9	B9	Sample 9	K9	—	—	—	—
10	Sample 10	B10	Sample 10	K10	—	—	—	—
11	Sample 11	B11	Sample 11	K11	—	—	—	—
12	Sample 12	B12	Sample 12	K12	—	—	—	—
13	Sample 13	B13	Sample 13	K13	—	—	—	—
14	Sample 14	B14	Sample 14	K14	—	—	—	—
15	Sample 15	B15	Sample 15	K15	—	—	—	—
16	Sample 16	B16	Sample 16	K16	—	—	—	—
17	Sample 17	B17	Sample 17	K17	—	—	—	—
18	Sample 18	B18	Sample 18	K18	—	—	—	—
19	Sample 19	B19	Sample 19	K19	—	—	—	—
20	Sample 20	B20	—	—	—	—	—	—

B: blue color; K: black color; R: red color; G: green color.

**Table 2:** DP for UV/Vis and FTIR of blue, black, red, and green ballpoint inks calculated by visual analysis.

Technique	DP (no. of groups)			
	Blue (*n* = 20)	Black (*n* = 19)	Red (*n* = 8)	Green (*n* = 6)
UV/Vis	0.563 (3)	0.812 (5)	0.678 (3)	0.866 (4)
FTIR	0.605 (4)	0.444 (4)	0.642 (3)	0.866 (4)

UV/Vis: UV/visible spectroscopy; FTIR: Fourier transform infrared spectroscopy.

**Table 3:** Cumulative variance (%) explained by PCA of ballpoint pen inks.

	Cumulative variance (%)	
	Cumulative variance explained by the first 2 principal components	
Ink color	FTIR spectroscopy	UV/Vis spectroscopy
Blue	94.227	98.872
Black	95.787	98.519
Red	98.893	99.092
Green	96.935	98.197

FTIR: Fourier transform infrared spectroscopy; UV/Vis: ultraviolet visible spectroscopy.

**Table 4:** The calculations for the number of clusters and DP for each cluster achieved from UV/Vis spectroscopy.

UV/Vis spectroscopy	ID of cluster	No. of ballpoint samples in cluster	Samples in cluster	Nondiscriminating sample pairs in cluster	Total no. of sample pairs	No. of discriminating sample pairs	DP	Average DP (for 2 clusters)
Blue	1	8	1, 3, 4, 5, 6, 9, 14, 18	—	28	28	1	0.98
	2	12	2, 7, 8, 10, 11, 12, 13, 15, 16, 17, 19, 20	12, 13 and 19, 20	66	64	0.969	

Black	1	8	1, 2, 4, 5, 6,7, 11, 13	—	28	28	1	0.99
	2	11	3, 8, 9, 10, 12, 14, 15, 16, 17, 18, 19	12, 14	55	54	0.98	

Green	1	4	1, 3, 4, 6	—	6	6	1	1
	2	2	2, 5	—	1	1	1	

Red	1	5	1, 3, 4, 7, 8	—	10	10	1	1
	2	3	2, 5, 6	—	3	3	1	

UV/Vis: ultraviolet visible spectroscopy; DP: discriminating power.

**Table 5:** DP calculations of ballpoint pen inks with cluster analysis.

Color of ballpoint pen	DP with UV/Vis data cluster analysis	DP with FTIR data cluster analysis
Blue	0.98	0.99
Black	0.99	1
Red	1	1
Green	1	1

DP: discriminating power; UV/Vis: ultraviolet visible spectroscopy; FTIR: Fourier transform infrared spectroscopy.

**Table 6:** The calculations for the number of clusters and DP for each cluster achieved from FTIR spectroscopy.

FTIR spectroscopy	ID of cluster	No. of ballpoint samples in cluster	Samples in cluster	Nondiscriminating sample pairs in cluster	Total no. of sample pairs	Discriminating sample pairs	DP	Average DP (for 2 clusters)
Blue	1	8	1, 2, 3, 7, 8, 9, 14, 19	—	28	28	1	0.99
	2	12	4, 5, 18, 6, 10, 11, 12, 13, 15, 16, 17, 20	5, 18	66	65	0.98	

Black	1	10	1, 2, 6, 11, 12, 13, 14, 16, 17, 19	—	45	45	1	1
	2	9	3, 4, 5, 7, 8, 9, 10, 15, 18	—	36	36	1	

Green	1	4	1, 2, 3, 5	—	6	6	1	1
	2	2	4, 6	—	1	1	1	

Red	1	3	1, 2, 7	—	3	3	1	1
	2	5	3, 4, 5, 6, 8	—	10	10	1	

FTIR: Fourier transform infrared spectroscopy; DP: discriminating power.

**Table 7:** Comparison of discrimination for the current study and previously reported studies in the literature.

Serial. no. with references	Total no. of samples for ballpoint inks	Used instrument	Used methods	Analysis type	Conclusions
A [11]	33 (21 black, 12 blue ballpoint pen)	UV/Vis, thin layer chromatography, and FTIR	Destructive analysis	Destructive	100% for black, 98% for blue ink

B [16]	08 blue ballpoint pen	High-pressure liquid chromatography and FTIR	PCA and LDA	Destructive/nondestructive	97.9%

C [36]	21 blue ballpoint pen	LA-ICP-MS	MANOVA, Tukey's HSD and T2 Hoteling	Destructive	100% discrimination in different brands and partial discrimination in same bands

D [10]	10 black ballpoint pen	Luminescence spectroscopy	Principal component analysis	Nondestructive	87% discrimination at 95% confidence interval

E [13]	41 blue ballpoint pen	Thin layer chromatography and image analysis	RGB Profiles	Destructive	92.8%

F [37]	57 blue ballpoint	UV/Vis and UV/Vis -NIR	Principal component analysis	Destructive and nondestructive	98.72% destructive 99.46% nondestructive

G [3]	57 blue ballpoint	HPTLC and FTIR	Principal component analysis	Destructive and nondestructive	93.80% destructive 99.69% nondestructive

H (current research)	55 (20 blue, 19 black, 8 red, and 6 green ballpoint pens)	UV/Vis and FTIR	PCA and cluster analysis	Destructive	99% blue ink, 100% black, red, and green inks

FTIR: Fourier transform infrared spectroscopy; UV/Vis: ultraviolet visible spectroscopy.

## Data Availability

The data used to support the findings of this study are available from the corresponding author upon request.
